# Explore the Effect of Asthma Regulating HIF-1 Pathway on Sperm Quality Based on Rat Model

**DOI:** 10.1155/2022/4194685

**Published:** 2022-05-17

**Authors:** Junlong Feng, Yuan Tang, Zhen Yang, Binghao Bao, Yichen Liu, Sheng Deng, Haisong Li, Jiangbin Li, Jisheng Wang

**Affiliations:** ^1^Beijing University of Chinese Medicine, Beijing 100029, China; ^2^Department of Andrology, Dongzhimen Hospital, Beijing University of Chinese Medicine, Beijing 100700, China; ^3^Urology Andrology Center of Peking University First Hospital, Beijing 100034, China; ^4^Department of Andrology, Shunyi Hospital of Beijing Traditional Chinese Medicine Hospital, Beijing 101300, China

## Abstract

This study is to verify the effect of asthma on sperm quality and explore its potential underlying mechanism. We randomly categorized the Sprague-Dawley (SD) rats into control (Group C) and asthma model (Group M) groups. Rats in the asthma model group were induced allergic asthma by intraperitoneal injection of ovalbumin solution. We evaluated the sperm motility and sperm concentration. The expression of the Interleukin-6 (IL6), phosphorylation-signal transducer and activator of transcription 3 (p-Stat3), and hypoxia-inducible factor-1*α* (HIF-1*α*) proteins and mRNAs in the testicular tissue was detected by western blotting and RT-qPCR. Compared with group C, sperm concentration and sperm motility in group M rats were significantly decreased (*P* < 0.05). Meanwhile, compared with group C, the expression levels of IL6, Stat3, and HIF-1*α* proteins and mRNAs in group M rats were significantly increased (*P* < 0.05). Asthma can regulate the HIF-1 signaling pathway, promoting the expression of IL6, Stat3, and HIF-1*α* protein and mRNAs, so as to promote sperm apoptosis and ultimately causing male infertility.

## 1. Introduction

Asthma is a chronic inflammatory respiratory disease with high morbidity and mortality. At present, about 10% people are affected by asthma and the incidence rate is still rising [1, 2]. Asthma can lead to airway edema, inflammation, fibrosis, airway obstruction, reduced ventilation, and damage to alveolar capillaries. These conditions can cause pulmonary ventilation or ventilation disorders, resulting in insufficient oxygen supply to lung tissue [3]. Hypoxia is mediated by HIF, which has two subunits of HIF-1*α*/2*α* and 1*β* [4]. HIF-1*α* is a transcription factor that plays a crucial role in regulating the inflammatory and metabolic genes of mammalian cells. Recent research results show that HIF-1*α* is the key regulator of asthma inflammation [5]. Asthma can activate HIF-1 signaling pathway in vivo, which can promote inflammation and induce the activation of genes related to airway remodeling [6]. Hypoxia response and significant increase of HIF-1 can be observed in mouse models of acute asthma and chronic asthma, resulting in increased inflammatory cell infiltration, fibrosis, and airway remodeling [7].

Infertility has always been a problem of concern. According to the statistics of the World Health Organization, 50-80 million couples in the world are troubled by infertility, about 20%-30% of which are caused by male factors [8, 9]. The pathogenesis of male infertility is complex. Studies have found that the epididymal tissue under hypoxia will lead to the overexpression of HIF-1*α*, which will affect the maturation and capacitation of sperm in the epididymis [10, 11]. And in the state of hypoxia, the testicular temperature will increase, morphology change, intercellular space increase, spermatogenic epithelium shrink, and the number of sperm decrease significantly [12–14].

Therefore, we hypothesized that hypoxia caused by asthma activates HIF-1 signaling pathway, which affects sperm quality and leads to male infertility. The aim of this study is to use bioinformatics analysis and animal experiments to predict and verify the molecular pathways and targets of asthma-induced male infertility. We followed the methods of Wang et al. [15]. The research idea is shown in Figure 1.

## 2. Methods and Materials

### 2.1. Molecular Target Recognition

Using asthma and infertility as key words, we used the GeneCards database (https://www.genecards.org/) [16] to obtain the related targets of the two diseases. The targets of asthma and male infertility were overlapped, and the intersection target was taken as the potential target for further analysis.

### 2.2. Analysis of Protein-Protein Interaction (PPI) Network

We used the STRING database (https://STRING-db.org/) [17] to determine possible PPI between potential action targets, the protein species is set as “homo sapiens.” In order to improve the reliability of the data, the PPI network of potential targets was obtained by taking the combined score >0.4 as the screening standard.

### 2.3. Network Construction and Analysis

Cytoscape version 3.8.0 (https://cytoscape.org/) [18] was used to construct an asthma-male infertility-target network and PPI network. After network construction, we used cytoHubba, a plug-in of Cytoscape, to further analyze the PPI network to identify the key targets [19].

### 2.4. Enrichment Analysis of GO Function and KEGG Pathway

We introduced the common targets of asthma and male infertility into the functional annotation tool of the “Database for Annotation, Visualization and Integrated Discovery” (DAVID, https://david.ncifcrf.gov/, v.6.8) [20] for gene ontology (GO) enrichment analysis and described the function of target genes. Using the DAVID database for “Kyoto Encyclopedia of genes and genomes” (KEGG) pathway enrichment analysis, the biological processes and key signaling pathways of male infertility caused by asthma were obtained [21].

### 2.5. Experimental Animals

20 specific pathogen-free (SPF) grade male SD rats (4–5 weeks old; 200–220 g) were purchased from Speyford (Beijing) Biotechnology Co., Ltd. (License Number: SCXK Beijing 2016-0002; Beijing, China). Rats were raised in the SPF animal feeding room of Beijing University of Chinese medicine, with indoor humidity of 60% and temperature of 24°C. The animals were fed with deionized water and solid feed for 7 days. The experimental animal ethics committee of Beijing University of Chinese Medicine approved the experimental scheme (No. BUCM-4-201991053064).

### 2.6. Drugs and Reagents

Drugs and reagents used included the following: Ovalbumin (Sigma, A5503; MO, USA); Aluminium hydroxide gel (Pierce, 77161; SH, CN); BCA protein quantitative kit (Chinese British Institute of Biotechnology, SI-5700; BJ, CN); c-DNA Kit (Thermo, #1622; MA, USA); IL6 antibody (Bioss, bs-6309R; Woburn, MA, USA); p-Stat3 antibody (Bioss, bs-1658R; Woburn, MA, USA); HIF-1*α* antibody (Bioss, bs-20398R; Woburn, MA, USA); Compression atomizer (Omron, NE-C900; DL, CN); and Stainless steel cell sieve (Puyi Biotechnology, PY-0643; SH, CN).

### 2.7. Construction and Grouping of Asthma Model

After 7 days of normal feeding, 6 rats were selected as the blank control group according to the random number table method, and the other 14 rats were modeled. For the first 3 weeks, the blank control group was intraperitoneally injected with 1 m sterile normal saline every day. On days 0, 7, and 14, the rats in the asthma model group were injected with 1 ml containing 100 mg ovalbumin (OVA) and 10 mg aluminium hydroxide gel via the peritoneal route. From the 22nd day, the rats in the blank control group inhaled sterile saline through a compression atomizer at a rate of 0.2 ml/min for 30 min, while rats in the asthma model group were administered 1% OVA through atomization at a rate of 0.2 ml/min over a course of 30 min. Both groups underwent surgery once a day for 3 weeks. After 3 weeks, we assessed the rats in the asthma model group in terms of their behavior, presence of upright fur, shortness of breath, nose scratching, and incontinence, as described in previous studies [22]. At the same time, the pathological sections of rat lung were observed for model evaluation. Finally, 10 of the 14 rats were successfully modeled. Then, 6 asthma model rats were randomly selected as the model group (group M, *n* = 6), and the previous 6 normal rats were regarded as the blank control group (group C, *n* = 6).

### 2.8. Analysis of Semen Quality

Rats in each group were weighed and anesthetized using sodium pentobarbital (50 mg/kg via intraperitoneal injection). Next, the testicular and epididymal tissues were removed, weighed, and transferred into EP tubes containing normal saline. Epididymides were removed, weighed, and transferred to preheated normal saline (0.9%). We put the comminuted epididymal tissue in the abovementioned 0.9% normal saline and incubated it in a 37°C water bath for 5 min. A stainless steel cell sieve was used to repeatedly filter the sperm mixture. Next, the sediment was removed and 1 ml of sperm fixative was added and agitated to enhance mixing. Subsequently, the spermatozoa were counted using a cell counting plate. The observation methods were according to the standard of the World Health Organization: a total of 200 sperm from 10 visual fields were randomly selected, of which the forward swimming sperm was forward motile sperm, and the in situ motile sperm was nonforward motile sperm. Dividing the number of the above sperm by 200, the percentage of forward motile sperm and nonforward motile sperm was obtained, which was the total sperm motility. The 10 fields were randomly chosen and the number of sperm in 10 large squares was counted. The mean value was given as 10^6^/ml.

### 2.9. Hematoxylin and Eosin (HE) Staining and Johnsen Score Test

Testicular tissue was fixed in 4% formaldehyde [23], dehydrated with gradient ethanol, embedded in paraffin, and then cut along the horizontal axis to create sections of 4 *μ*m thickness. The tissue was treated with ethanol and xylene for 3 min, washed with tap water, and then treated with eosin for 2 min. After dehydration and drying, the tissue was observed under a light microscope. Ten seminiferous tubules were selected under the light microscope, and the development of rat seminiferous epithelial cells was evaluated according to the Johnsen 10-level scoring method. The scoring criteria are as follows: 1 point, no cells; 2 points, Sertoli cells only; 3 points, only spermatogonia, no spermatogenic cells; 4 points, 5 spermatocytes; 5 points, more than 5 spermatocytes; 6 points, 1 to 5 sperm cells; 7 points, more than 5 sperm cells, but no differentiation; 8 points, the presence of advanced sperm cells; 9 points, 1 to 5 sperm cells; and 10 points, more than 5 sperm cells.

### 2.10. Western Blotting

The testicular tissue was collected and weighed. Then, RIPA strong lysate was added to it and the sample was homogenized on an ice bath, followed by centrifugation, separation of the supernatant, and determination of the total protein content by using the BCA method. The separation and thickening gel were prepared, sample on the protein, after the completion of the sample, the glass plate was placed in the electrophoresis tank, and gel electrophoresis was carried out at a constant pressure of 80 V. After the bromophenol blue dissipated from the separation gel, the protein was transferred onto the PVDF film. Then, 5% skim milk powder was sealed at 1 h at room temperature, and the strip was cut based on the molecular weight of the target protein, followed by overnight treatment at 4°C with a single antibody (diluted at 1 : 1000), and the following day, the strips were rinsed in TBST solution thrice, before treatment with the secondary antibody at room temperature for 4 h (1 : 1000 dilution), washed thrice with TBST, and developed by chemiluminescence. The band gray value was quantified by the Image-Pro Plus software to calculate the relative expression of the protein.

### 2.11. RT-qPCR

The testicular tissue was added to a mortar, to which a small amount of liquid nitrogen was added, followed by quick grinding 3 times. After grinding, add 1 ml TRIzol reagent was introduced and the total RNA was isolated from the tissue. After the content was qualified, the RNA was converted to cDNA based on the reverse transcription kit operational requirements, and then, the target gene product was amplified under the following conditions: predenaturation at 95°C for 15 min, denaturation at 95°C for 10 s, annealing, and extension at 60°C for 30 s, 40 cycles. After the reaction, the CT value to 2^−Ct△△^ was calculated. The relative gene expression was analyzed via the CT formula. *β*-Actin gene was employed as endogenous reference. The sequence of primers is listed in Table 1.

### 2.12. Statistical Analysis

All data analyses employed SPSS 26.0. Continuous data are presented as mean ± standard deviation. For data with normal distribution, a *t*-test was employed, and for data with not normal distribution, the nonparametric test was employed. *P* < 0.05 was deemed as significant.

## 3. Results

### 3.1. Target Collection, Construction of PPI Network, and Topology Analysis

After collection, the 500 male infertility-related targets and the 500 asthma-related targets were obtained from GeneCards. Then, 81 overlapping targets were obtained after taking their intersection (Figure 2(a)). Next, the asthma-male infertility-target network is shown in Figure 2(b). And a PPI analysis was performed on these overlapping targets through the STRING database; we confirmed that all targets were associated with both asthma and male infertility and used Cytoscape to build a network (Figure 2(c)). According to the cytoHubba analysis, the top 10 targets were regarded as key targets (Table 2 and Figure 2(d)).

### 3.2. Pathway Enrichment Analysis Using the DAVID Database

Using DAVID v6.8, 28 targets were enriched and analyzed. We found that there were 412 biological processes, 43 cell components, 47 molecular functions, and 65 signal pathways. According to the *P* values, the analysis results of the top 5 biological functions and pathways were selected for display (Figures 3(a) and 3(b)).

### 3.3. Validation of the Asthma Model

The rats in the asthma model group exhibited anxiety, upright fur, shortness of breath, obvious abdominal breathing, nose scratching, and incontinence. None of the control rats exhibited any of these symptoms. HE staining showed that the airway structure of normal rats was basically normal, almost without inflammatory cell infiltration. In the model group, the airway wall of lung tissue was proliferated, there is a large number of inflammatory cell infiltration, airway epithelial structure was disordered, and small airway lumen was narrow (Figure 4(a)); Masson staining showed that the collagen deposition in the airway submucosa of the model group was higher than that of the normal group (Figure 4(b)).

### 3.4. Body Weight of Rats and Wet Weight of Testis and Epididymis

The body weight and wet weight of epididymis in group M were lower than that in group C (*P* < 0.05), but there was no significant difference in testicular wet weight between group M and group C (*P* > 0.05) (Table 3).

### 3.5. Analysis of Semen Quality

The sperm concentration in group C was significantly higher than that in group M (*P* < 0.05). Furthermore, the sperm motility of group C was significantly higher than that of group M (*P* < 0.05, Table 4).

### 3.6. HE Staining of Testicular Tissue and Spermatogenic Cell Development Score

The seminiferous tubules in group C rats were normally structured and orderly arranged, and a large number of normal sperm and spermatogenic cells of all levels could be seen in the lumen. The cell structure in each layer was complete, orderly, clear, and with no obvious morphological abnormality (Figure 5(a)). In group M, the seminiferous tubules were abnormally structured and irregularly arranged. The lumen of the seminiferous tubules was contracted, the epithelium was degenerated partially. Moreover, the proportion of abnormal sperm increased significantly. The number of spermatozoa was significantly less (Figure 5(a)). Moreover, compared with group C, the development score of spermatogenic cells in group M was significantly lower (*P* < 0.05). The results are shown in Table 5.

### 3.7. Expression of IL6, Stat3, p-Stat3, and HIF-1*α* in Testicular Tissue Was Detected by Western Blotting

After 4 weeks of successful modeling, the protein expressions of IL6, Stat3, p-Stat3, and HIF-1*α* in group M were significantly lower than those in group C (*P* < 0.05) (Figures 5(b) and 5(c)).

### 3.8. mRNA Expression of IL6, Stat3, and HIF-1*α* in Testicular Tissue Was Detected by RT-qPCR

Compared with group C, the mRNA expression levels of IL6, Stat3, and HIF-1*α* in group M were significantly increased (*P* < 0.05) (Figure 5(d)).

## 4. Discussion

Our experimental results are consistent with the original hypothesis. The hypoxic environment caused by asthma activates HIF-1 signaling pathway, which affects sperm quality and leads to male infertility. At present, there are few studies on male infertility caused by asthma, and its potential mechanism is not clear. Here, we propose possible mechanism hypotheses through bioinformatics and animal experiments.

In this study, we found that the sperm concentration and sperm motility in group M were significantly lower than that in group C. In addition, HE staining showed that the lumen of seminiferous tubules in the testis of asthma model group was contracted, and the proportion of abnormal sperm and spermatogenic cells increased significantly. These results provide direct evidence that asthma may lead to male infertility.

Through the pathway enrichment analysis of network pharmacology, we found that HIF-1 signaling pathway is the key pathway of infertility caused by asthma. Hypoxia can induce a series of physiological and pathological reactions, such as accelerating energy metabolism and cell apoptosis, promoting angiogenesis and remodeling, these reactions are mainly mediated by HIF-1 [24]. Research shows that IL6 and Stat3 are HIF-1*α* important upstream signal genes [25], and IL-6/Stat3/HIF-1*α* signaling pathway plays an important role in many diseases. IL-6 plays a role by binding to IL-6 receptor (IL-6R). After the two combine to form a complex, they contact with signal transduction membrane protein gp130, the receptor dimerization occurs, and the IL-6 signal transduction pathway is activated. The downstream Stat3 can be further activated by activating JAK2, and the activated Stat3 can block hypoxia induced HIF-1*α* degrading or promote its synthesis, so as to improve HIF-1*α* expression level [26, 27].

IL6 is a multiactive cytokine, which can promote the proliferation and differentiation of a variety of cells. It is found that Th17 cells play an important role in inducing chronic airway inflammation. IL6 can promote the differentiation and proliferation of Th17 cells and aggravate airway inflammatory response by inhibiting macrophages [28, 29]. Moreover, IL6 plays an important role in the male reproductive system because it can reduce sperm penetration, antioxidant activity, reduce sperm parameters, and cause long-term inflammation of the male reproductive system [30]. Stat3 is a cytokine-activated transcription factor, and its activation plays a key role in regulating inflammatory response. Once stimulated, it leads to the phosphorylation of Stat3 Tyr705 site and is then transferred to the nucleus, thus transcriptionally regulating the production of cytokine response genes and cytokines [31]. Activation of Stat3 can also promote the production of Th2 and Th17 cytokines promote inflammatory response, and aggravate asthma [32]. Studies show that Stat3 protein can regulate the differentiation and proliferation of spermatogonial stem cells during mammalian spermatogenesis and can affect the apoptosis process of spermatogonia and spermatocytes at all levels (including primary and secondary spermatocytes) [33, 34]. In the pathogenesis of asthma, with the activation of IL6 and Stat3 proteins, HIF-1*α* protein expression increases under the IL-6/Stat3/HIF-1*α* signaling pathway, which then promotes the apoptosis of spermatogenic cells, affecting sperm quality [35]. Our experimental results showed that the expression of IL6, Stat3, and HIF-1*α* increased significantly in the asthma model group, and the sperm concentration and total sperm viability decreased significantly in the model group, which proved that asthma could increase the expression of IL6, Stat3, and HIF-1*α* protein, promote the apoptosis of spermatogenic cells, and lead to infertility.

The relationship between asthma and male infertility is rarely discussed in the literature. Therefore, this study adopts a new method to explain the basic mechanism of male infertility caused by asthma through biological network analysis and experimental verification in rat model, in order to provide some guidance for clinical treatment in the future. Of course, our article also has shortcomings. For example, we did not measure sex hormones in rats. It has been found that hypoxia caused by asthma can also lead to endocrine dysfunction and affect sperm motility [36]. Moreover, we lack cell experimental verification of low/overexpression of HIF-1 and further detection of apoptotic factors. In the future research, we will optimize the experimental scheme and further explore the causes of spermatogenesis dysfunction caused by asthma, so as to provide new theories and schemes for clinical diagnosis and treatment.

## 5. Conclusion

This study shows that asthma can regulate the HIF-1 signaling pathway, promoting the expression of IL6, Stat3, and HIF-1*α* protein and mRNAs, so as to promote sperm apoptosis and ultimately causing male infertility.

## Figures and Tables

**Figure 1:** Overall process based on biological network research and animal experiments.

**Figure 2:** (a) Intersection of targets of asthma and male infertility. (b) Asthma-male infertility-target network built by Cytoscape (3.7.1). (c) PPI network built by Cytoscape (3.7.1). (d) PPI network processed by Cytoscape (3.7.1) plug-in (cytoHubba).

**Figure 3:** (a) GO enrichment analysis: the length of the bar is related to the number of enriched genes. (b) KEGG enrichment analysis: *x* axis represents rich factor, *y* axis represents name, node size is related to count, and node color is related to *P* value.

**Figure 4:** (a) HE staining of lung tissue in two groups. (b) Masson staining of lung tissue in two groups.

**Figure 5:** (a) Analyses of testicular tissue in mice using HE staining. (b) Electrophoretogram of three proteins (IL6, Stat3, p-Stat3, and HIF-1*α*) in rats from the C, M groups. (c) The expression levels of three proteins (IL6, Stat3, p-Stat3, and HIF-1*α*) in rats from the C, M groups determined using western blotting. (d) The mRNA expression levels of three proteins (IL6, Stat3, and HIF-1*α*) in rats from the C, M groups determined using RT-qPCR. Values are the mean ± SEM (*n* = 6 animals per group). The *t*-test was used. Group M was compared with group C, ^∗^ represents *P* < 0.05, ^∗∗^ represents *P* < 0.01.

**Table 1:** The primer sequences for RT-qPCR.

Primer	Forward	Reverse
IL6	5′-CTCACGCACCGATGTCT-3′	5′-AGGCTGTGGGCTCAATC-3′
Stat3	5′-GGAGGAGGCATTCGGAAAG-3′	5′-TCGTTGGTGTCACACAGAT-3′
HIF-1*α*	5′-ACAAGCCACCTGAGGAGAGG-3′	5′-TGGCTGCATCTCGAGACTTT-3′
*β*-Actin	5′-GCACTCTTCCAGCCTTCCTT-3′	5′-AATGCCAGGGTACATGGTGG-3′

**Table 2:** Top 10 key targets.

Rank	Target name	Score
1	Tumor necrosis factor (TNF)	65
2	Albumin (ALB)	63
3	Glyceraldehyde-3-Phosphate Dehydrogenase (GAPDH)	59
3	Interleukin 6 (IL6)	59
5	Insulin (INS)	58
6	Vascular endothelial growth factor A (VEGFA)	57
7	Interleukin 1 beta (IL1B)	55
8	Epidermal growth factor receptor (EGFR)	51
9	Interleukin 10 (IL10)	50
10	C-X-C motif chemokine ligand 8 (CXCL8)	48

**Table 3:** Body weight of rats and wet weight of testis and epididymis. *g*, *n* = 6,$\bar{x}\pm s$.

Group	Body weight of rats	Wet weight of testis	Wet weight of epididymis
Group C	263.83 ± 6.09	3.12 ± 0.12	1.08 ± 0.03
Group M	223.47 ± 9.46^∗^	3.02 ± 0.14	0.96 ± 0.02^∗^

Note: Differences with *P* < 0.05 were considered statistically significant. ^∗^*P* < 0.05 vs. Group C.

**Table 4:** The sperm concentration and sperm motility of rats from the C, M groups.10^6^/ml, %, *n* = 6, $\bar{x}\pm s$.

Group	Sperm concentration	Sperm motility
Group C	44.29 ± 5.50	59.68 ± 4.84
Group M	14.20 ± 1.65^∗^	16.92 ± 2.99^∗^

Note: Differences with *P* < 0.05 were considered statistically significant.^∗^*P* < 0.05 vs. Group C.

**Table 5:** Spermatogenic cell development scores of rats in each group. *n* = 6, $\bar{x}\pm s$.

Group	Johnsen score
Group C	9.67 ± 0.58
Group M	6.33 ± 0.57^∗^

Note: Differences with *P* < 0.05 were considered statistically significant. ^∗^*P* < 0.05 vs. Group C.

## Data Availability

The data that support the findings of this study are available from the corresponding author upon reasonable request.
